This article has been retracted.

# Analysis of the Overall Development Mode of Cultural Tourism under the Creative Economy Environment

**DOI:** 10.1155/2022/3498622

**Published:** 2022-09-14

**Authors:** Hongrui Zhang

**Affiliations:** School of Tourism, Shandong Women's University, Jinan Shandong 250300, China

## Abstract

Tourism is evolving constantly as a result of the growth of the creative economy. Currently, ethnic cultural tourism is the focus of cultural tourism's overall development, while cultural tourism's development is primarily driven by considerations of social economy, cultural protection, and cultural inheritance. The first section of the article defines cultural and creative tourism. Second, this essay examines the evolution of creative and cultural tourism in general. In the end, cultural tourism's overall development is unquestionably superior to other development, and the other two commonly receive poor ratings. Its overall development score ranges from 4.4 to 4.9, and its average value without overall development is 4.42. The highest score is 4.89, with the average for cultural tourism with limited development being 4.49 and the average for cultural tourism with full development being 4.71. In a nutshell, the paper's proposal for evaluating the entire development of cultural tourism is doable.

## 1. Introduction

Creativity is a kind of productive force composed of immaterial factors such as imagination, concept, culture, and emotion [1]. It has unlimited imagination space. It can promote innovation through imagination, sublimate ideas into values, create selling points for culture, and transform emotions into market advantages, thereby promoting changes in production methods and lifestyles. Many cultural development practices in today's world show that in terms of knowledge, intelligence, technology, etc., especially in knowledge, intelligence, technology, etc., it is more diverse and richer than the general manufacturing and service industries, and it is an imaginative and creative industry field [2]. “Cultural tourism” is a new concept that has emerged in recent years, and its emergence is closely related to the changes in tourists' needs [3]. Therefore, the more popular definition now is cultural heritage, architecture, national art, folk customs, religion, and other aspects of tourism.

The concept of “creative economy” is constantly emerging and gradually accepted by the public. The basic idea of innovation economy is to take innovation and culture as the center, and promote the integration and cooperation of industries through the boundaries of cross-organizations [4]. In the modern service industry, many sectors intersect with tourism. China's tourism industry is facing new challenges under the environment of innovative economy [5]. China's tourist sector has entered the period of mass tourism from the standpoint of industry development, but the growth of the entire industry is still relatively sluggish as a result of its excessive reliance on elements like nature and the environment. Emphasizing the extensional development of material components while ignoring the investment in nonmaterial aspects is what propels tourist development. As a result, the cultural relevance and knowledge of innovation of tourism products are insufficient. The “creative turn” concept has risen in popularity as a result of the conflict between the development of new cultural tourism items and the issue of cultural duplication [6]. In light of the creative economy, this essay suggests conducting research on the general development model of cultural tourism. The collaborative filtering algorithm and association rules are used to lessen the impact of subjective factors on the overall growth and evaluation of cultural tourism, as well as to mine potential factor associations during the evaluation process. This algorithm support will help establish a more rigorous and objective tourism evaluation system and will improve the objectivity of evaluation techniques. Additionally, the reliability of the evaluation's findings is important for the development of cultural tourism research as a whole.

Breaking free from the constraints of tradition and fostering the optimization and upgrading of the industrial structure based on greater knowledge are made possible by the mix of tourism, cultural, and creative industries [7]. Tourism, cultural, and creative industries will inevitably flourish together in the context of the creative economy. The National Tourism Administration has advocated vigorously for the transformation and upgrading of the tourism industry in recent years, from extensive development to intensive development, from focusing on scale expansion to giving equal attention to expanding scale and improving efficiency, and from focusing on economic functions to fully embracing comprehensive functions [8]. The innovation of tourism mode is an inevitable choice for the transformation and upgrading of the tourism industry [9]. From the point of view of systems theory, industrial convergence is essentially the adaptive choice of industrial systems to dynamic environments. The emergence of industrial integration has made the industry with clear industry boundaries to form a new industrial form in the integration of industrial boundaries and has become an important value growth point and a source of power for economic growth [10]. The main contributions of this paper are as follows:

1. In this paper, the collaborative filtering algorithm and association rule algorithm are used to construct the evaluation and evaluation model in the overall development of cultural tourism
2. This text research will use a variety of related research methods to compare, so as to obtain comprehensive and in-depth research results on this topic and promote the effect of the overall development of cultural tourism

## 2. Related Work

Cultural tourism refers to the viewing and recreational forms created by tourists as consumption content so that tourists can get rich cultural connotations in tourism and can better participate in tourism. Cultural tourism is a kind of tourism with the main purpose of appreciating foreign cultures, pursuing cultural celebrity relics, and participating in cultural activities in various places. The pursuit of cultural enjoyment has become a fashion for today's tourists [11]. Cultural tourism is not only a commodity but also a distinct product from mainstream tourist. Tourism is merely a “form,” whereas the so-called “culture” is “culture.” “Culture” is a description of how and why tourism-related activities are used. In general, regardless of whether the excavation process considers consumer demand and competition, it looks for variations and characteristics from the perspective of resources. In a way, resources, environment, market, and social background, or “creativity,” can all be combined to create cultural tourism. Cultural tourism will not thrive if it lacks inventiveness. As a result, only tourism products that place a strong emphasis on cultural originality may really satisfy the psychological and emotional needs of contemporary travellers.

Ardissono et al. adopted the virtual reality development technology Unity3D and produced the Nanyin cultural interactive tourism system, which enhanced the viewer's sense of immersion and experience [12]. Wang et al. used Arc GIS Engine technology to realize the cultural tourism system of colleges and universities, showing the cultural characteristics of the campus [13]. Ma developed a cultural tourism system with the help of UAV aerial photography, GIS, and other technologies, providing strong support for the tourism industry [14]. Wen discussed the products and consumption of European cultural tourism, arguing that although the demand for heritage tourism is on the rise with the increase of tourists' income and education, the change in demand is more affected by supply [15]. At the same time, the production of heritage tourism products is limited in space, and the consumers of heritage tourism products are mainly some new middle class with limited consumption, so it is difficult to increase tourism supply. Bui and Trupp illustrates that museums with educational and cultural functions play an increasingly important role in urban economic development and tourism development [16]. Dong et al. discussed the cultural heritage of the community and its importance, conducted random questionnaire surveys and interviews with local residents, and processed the results through the factor analysis method of SPSS, proposed a tourism development model, and used tourism centers [17]. And peripheral center concepts are explained to guide regional tourism planning. Ridwan studied the development stages of heritage tourism and its authenticity, arguing that the authenticity of heritage tourism resources is a determinant of product quality and tourist satisfaction [18]. Liu analyzed the cultural factors and community participation factors in the development of rural cultural tourism, explored a mode of rural cultural tourism development, and emphasized the importance of rural tourism culture [19]. Niels et al. adopted a decision tree-based algorithm to learn user preferences and recommend movies and news to users [20]. Calvillo et al. proposed a personalized recommender system integrating clustering and two mining techniques, a recommendation model for e-learning websites [21].

In the context of the creative economy, if the integrity of tourist attractions is not taken into account or due to the increase in the number of local attractions, more tourists will result. From the perspective of cultural tourism, the research on cultural tourism mostly focuses on heritage tourism, cultural tourism products, community participation, and government behavior. Therefore, this paper will use collaborative filtering algorithm and association rules to study the overall development model of cultural tourism in the context of creative economy.

## 3. Methodology

### 3.1. The Basic Concept of Cultural Tourism under the Creative Economy and Its Analysis

The cultural and creative tourism complex is a new form of tourism that has not yet developed a distinct and cohesive notion in domestic academic circles. Urban complexes, tourist complexes, and innovative tourism complexes are all closely related. A multipurpose and highly effective facility that includes commercial shops, office space, a hotel and catering, extensive entertainment, and apartments is referred to as a complete commercial complex. A tourist complex is a tourism and leisure community with high-quality complete services built on specific tourism resources and land, through comprehensive tourism and leisure development, with resort hotels, extensive leisure projects, and leisure real estate communities as the core. The tourism complex has seen numerous stages of development, with each stage's development focus being distinct, before finally becoming a particular gathering and scale. Additionally, one of them is the effect of tourism promotion (Figure 1).

In the context of the integration of tourism with cultural and creative industries, the term “cultural and creative tourism complex” refers to a new tourism business created by merging it with the six components of tourism (food, accommodation, transportation, travel, shopping, and entertainment). In the actual world, we may combine different travel experiences in a variety of ways to produce fresh, original encounters. Complexes that focus on culture and creativity as their “core” include a variety of social, economic, cultural, aesthetic, and geographical qualities and are well suited to satiating visitors' requirements for information, culture, the arts, and other pursuits. Optimizing the industrial structure of the tourism industry, expanding the industrial chain, fostering industrial transformation, and boosting the influence and driving power of the tourism industry are all possible with the creation of a cultural and creative tourism complex.

Its characteristics are as follows:

1. High degree of integration: cultural and creative tourism complex is a combination of tourism and cultural and creative industries, and it is a new form of tourism that crosses industry boundaries
2. Be creative: “creativity” is the core of cultural and creative tourism complex, and tourism products and services are the crystallization of human knowledge, wisdom, and inspiration, and the uniqueness of creativity is an important factor affecting its sustainable development
3. Very cultural: cultural and creative tourism complexes focus on the exploration and dissemination of culture, so that tourists can feel the charm and connotation of its culture in the in-depth development

Culture is divided into broad and narrow senses. In a broad sense, culture refers to “material and spiritual wealth produced in the historical process of human social development,” while “culture” in a narrow sense refers to “the corresponding social system and organizational structure.” How does culture transform into cultural industry? The industrialization process of culture includes three levels: commercialization, organization, and scale (Figure 2).

### 3.2. Text Representation Model

Information in nature cannot be recognized by computers, and they need to use the expression technology of words to convert unrecognizable, unrecognizable, structured, recognizable, and structured sentences. In many applications, the expression of text is necessary, such as extracting user sentiment from news topics, extracting sentiment from user product reviews, intelligent question answering systems, etc. Therefore, it is very necessary to extract the features of the text. There are two main methods for extracting text features: vector space and topic.

#### 3.2.1. Vector Space Model

The vector space model means that each document can be represented as a vector in the space. The features of the text can be expressed as

(1) $$\begin{array}{c} d=\left(t_{1},t_{2},t_{3},\cdots ,t_{n}\right). \end{array}$$

The weight corresponding to each feature can be expressed as (*w*_1_, *w*_2_, *w*_3_, ⋯, *w*_*n*_); therefore, the entire text can be expressed as a text containing feature weights as follows:

(2) $$\begin{array}{c} d=\left(t_{1},w_{1},t_{2},w_{2},t_{3},w_{3},\cdots ,t_{n},w_{n}\right). \end{array}$$

At this time, the similarity between vectors can be equivalently expressed as the similarity between texts, as shown in Figure 3.

*D*_1_ and *D*_2_, respectively, represent two documents, (*w*_11_, *w*_12_, *w*_13_, ⋯, *w*_1*n*_) which are the feature vectors corresponding to the first document and the feature vectors corresponding (*w*_21_, *w*_22_, *w*_23_, ⋯, *w*_2*n*_) to the second document. But

(3) $$\begin{array}{c} D_{1}=d_{1}\left(w_{11},w_{12},w_{13},\cdots ,w_{1n}\right), \end{array}$$

(4) $$\begin{array}{c} D_{2}=d_{2}\left(w_{21},w_{22},w_{23},\cdots ,w_{2n}\right). \end{array}$$

To express the similarity between them, the cosine formula of the following vector can be used:

(5) $$\begin{array}{c} \text{similarity}=\cos\left(\theta \right)=\frac{A•B}{\left|\left|A\right|\right|•\left|\left|B\right|\right|}=\frac{\sum_{i=1}^{n}A_{i}\times B_{i}}{\sqrt{\sum_{i=1}^{n}{\left(A_{i}\right)}^{2}}\times \sqrt{\sum_{i=1}^{n}{\left(B_{i}\right)}^{2}}}. \end{array}$$

#### 3.2.2. Theme Model

Topic model is a mathematical model based on text semantic analysis and mining, and it is a representative unsupervised learning method. PLSA mode is also called PLSI mode, namely PLSI mode. Each article generally includes several topics, but their weights are different. There are several words under each topic, and each has a different weight. Below, represented by a few mathematical symbols are as follows:

1. Document collection

(6) $$\begin{array}{c} d=\left(d_{1},d_{2},d_{3},\cdots ,d_{n}\right). \end{array}$$

(2) The collection of words

(7) $$\begin{array}{c} w=\left(w_{1},w_{2},w_{3},\cdots ,w_{n}\right). \end{array}$$

(3) Theme collection

(8) $$\begin{array}{c} z=\left(z_{1},z_{2},z_{3},\cdots ,z_{n}\right). \end{array}$$

So

(9) $$\begin{array}{c} p\left(w_{j}\left|d_{i}\right.\right)=\overset{K}{\underset{k=1}{\sum }}p\left(w_{j}\left|z_{k}\right.\right)p\left(z_{k}\left|d_{i}\right.\right). \end{array}$$

Since the *p*(*w*_*j*_|*d*_*i*_) document-word matrix is known and can be obtained by calculating the text, what is needed in this paper is the text-topic matrix and the topic-word matrix, and the EM algorithm is used to solve the parameters.

### 3.3. Collaborative Filtering Algorithm

The core of the collaborative screening algorithm is collaboration, that is, to provide similar samples to the target samples. Collaborative filtering algorithms mainly include user collaboration and project collaboration. For example, according to the collaborative screening of products, since the user's evaluation of the product is a sparse matrix, many users' evaluation of the product is unclear. Therefore, we need to determine whether the user has evaluated a certain product, that is, the rating of this item and the similarity between this item. Finding similarities in similar samples is called collaborative screening. On the basis of the traditional cooperative filtering algorithm, an algorithm based on machine learning and a CNN algorithm based on deep learning are proposed. This section will detail two common collaborative filtering algorithms.

According to the collaborative filtering algorithm of the target user, it is according to the user's preference and users who use the same object who must have the same preference, so the same product can be recommended to the user. For example, users are matched according to their favorite travel locations, as shown in Figure 4.

When calculating the similarity between statistical samples, there are mainly four methods of similarity statistics, which are the Euclidean distance method, cosine similarity, Pearson similarity, and Jaccard similarity.

1. Euclidean distance method uses the distance formula. The smaller the distance, the higher the similarity. The formula is as follows:

(10) $$\begin{array}{c} \rho =\sqrt{{\left(x_{2}-x_{1}\right)}^{2}+{\left(y_{2}-y_{1}\right)}^{2}}. \end{array}$$

(2) Cosine similarity: in order to represent how similar two sides are, the cosine similarity is calculated by finding the cosine value of the angle between the two sides

(11) $$\begin{array}{c} \cos\left(\theta \right)=\frac{A•B}{\left|\left|A\right|\right|•\left|\left|B\right|\right|}=\frac{\sum_{i=1}^{n}A_{i}\times B_{i}}{\sqrt{\sum_{i=1}^{n}{\left(A_{i}\right)}^{2}}\times \sqrt{\sum_{i=1}^{n}{\left(B_{i}\right)}^{2}}}. \end{array}$$

(3) Pearson similarity is actually an improved cosine similarity, but the user's ratings are centralized in order to unify the rating system. The formula is as follows:

(12) $$\begin{array}{c} r=\frac{\sum_{i=1}^{n}\left(X_{i}-\bar{X}\right)\left(Y_{i}-\bar{Y}\right)}{\sqrt{\sum_{i=1}^{n}{\left(X_{i}-\bar{X}\right)}^{2}}\sqrt{\sum_{i=1}^{n}{\left(Y_{i}-\bar{Y}\right)}^{2}}}. \end{array}$$

(4) Jaccard similarity is also applied to Boolean vectors and refers to the percentage of the intersection of two sets in their union. The formula is as follows:

(13) $$\begin{array}{c} J\left(A,B\right)=\frac{\left|A\cap B\right|}{\left|A\cup B\right|}. \end{array}$$

### 3.4. Association Rules

The representation of *X*⟶*Y* association *X* rules is called the predecessor in the *Y* association rule and the successor in the association rule. The meaning of expressions refers to *X* the laws that appear at the same time as they appear *Y*.

Item, itemset: an item is an object we study, an itemset is a collection of single or multiple objects, and objects in an itemset cannot be repeated. Let *I* = {*i*_1_, *i*_2_, *i*_3_, ⋯*i*_*n*_}be *n* itemset containing items, where *i*_*k*_ is an item and *I* is *n*− itemset.

Support: support refers to how often an item occurs in a dataset. The greater the support, the greater the probability that the event will occur.

(14) $$\begin{array}{c} \text{support}\left(A\right)=\frac{\text{count}\left(A\right)}{\text{count}\left(\text{dataset}\right)}=P\left(A\right). \end{array}$$

Confidence: confidence is the number of times the item *A* co *B*-exists with the item, divided by the number of items that only contain *A* the item. It can be understood as *A* the probability that the user buys the product under the premise that he buys the product. *B* The meaning of the confidence is: when the confidence is very large, it means that when a user buys *A*, he has a high probability to buy *B*, then it *A* will make a lot of sense for us to bundle and sell. *B* If the confidence level is very low, it means that when the user purchases *A*, *B* the probability of purchase is very low, then this association rule is meaningless. Therefore, confidence reflects whether an association rule can reflect value.

(15) $$\begin{array}{c} \text{confidence}\left(A⟶B\right)=\frac{\text{count}\left(AB\right)}{\text{count}\left(A\right)}=\frac{\text{count}\left(AB\right)/\text{count}\left(\text{dataset}\right)}{\text{count}\left(A\right)/\text{count}\left(\text{dataset}\right)}=\frac{P\left(AB\right)}{P\left(A\right)}=P\left(B\left|A\right.\right). \end{array}$$

## 4. Result Analysis and Discussion

The research object of this paper is Yichun Scenic Area. Yichun is located in the northwest of Jiangxi Province, next to Feng City, Gao'an City, Yuanzhou District, Zhangshu City, Jing'an County, Fengxin County, Shanggao County, Yifeng County, Tonggu County, and Wanzai County. The land area is 1.8700 square kilometers, accounting for 11.20% of the country; the national population is 5.53 million, ranking second in the province, after Shangrao and Ganzhou.

Terrain condition: located at the junction of mountains and plains, the terrain is higher, and the terrain is lower. Among them, mountains and hills make up 39.10% and 25.77% are plains.

Climate characteristics: a typical subtropical region, with mild climate and abundant rainfall. There are distinct four seasons, spring, autumn, summer and winter. The city's annual average temperature is 17.2°C. It is hot in summer and above 0°C in winter, up to more than 9 months.

Hydrological resources: there are abundant groundwater and mineral water in every county and urban area.

Natural resources: *Camellia oleifera*, tung oil, soybean, ramie, ranking first in the country; rich underground reserves, mainly rare metals; water energy, wind energy, and light energy are the main sources of energy.

The division of its scenic spots (Table 1) and its tourist attractions (Table 2) are as follows.

The first part is the main part, which tests the evaluation of 15 perceptual elements (indicators at the index level).

The experimental results show that the overall development evaluation model of cultural tourism using collaborative filtering algorithm and association rules can evaluate and predict multiple data sets, respectively, and obtain exact data. From Figures 5 and 6, the number of people with each rating basically exists. Tourists have different concepts and ideas about the overall development of cultural tourism. However, it can be seen that most tourists score at 3 points, and there are still many tourists who are interested in cultural tourism. The overall development of tourism maintains a good attitude, giving 5 points. Elements 9–12 have a relatively large impact, that is, the theme of the cultural scenic spot, the industry of the cultural scenic spot, and the attractiveness of the cultural scenic spot.

In addition, this paper extracts user comments on Yichun scenic spot, and makes a chart, as shown in Figure 7 and Table 3.

From the chart, tourists still pay great attention to the influence of culture on the overall development model of tourism. The confidence value of “cultural teaching” is as high as 0.9, the value of historical significance is as high as 0.98, and the frequency of appearance of characteristic features in other tourists' visits. It is also conducive to the overall development of cultural tourism.

Yichun Zen cultural tourism, including cultural value, brand image, tourism products, cultural dissemination, tourism interpretation system, and tourists' participation, are finally transformed into an independent variable, and tourists' loyalty is the dependent variable. Partial development and overall development of cultural tourism are compared. Finally, from Figure 8, it can be seen that the overall development of cultural tourism is obviously better than other developments. The average is 0.78, the best of which can be as high as 0.96 for loyalty.

Figure 9 shows that the six dimensions of Zen cultural tourism, including cultural value, brand image, tourism products, cultural dissemination, tourism interpretation system, and tourist participation, are transformed into an independent variable, and tourist satisfaction is the dependent variable. The overall development, the implementation of partial development, and the implementation of overall development of cultural tourism will be self-scoring. It can be concluded that the overall development of cultural tourism has a much better effect than other developments, and the other two frequently have low scores, while the overall development of cultural tourism has a score of 4.4–4.9, and the average value of cultural tourism without overall development is 4.42, the average of cultural tourism with partial development is 4.49, the average of cultural tourism with overall development is 4.71, and the highest score is 4.89. In a word, the final effect evaluation of the overall development of cultural tourism proposed in this paper is feasible.

## 5. Conclusion

The overall development of cultural tourism is the dominant form of tourism in the future, and there are differences between the overall development of cultural tourism and other tourism development, because the regional culture of the destination is a whole, only through the overall development can it fully display its characteristics and maintain the long-term inheritance of culture. From the perspective of cultural form and structure and the level of tourism aesthetics, the concept and mode of overall development of cultural tourism are proposed, which have important theoretical and practical significance. Tourism and cultural and creative industries are both important components of modern service industries; these are the two major industries. The integration of tourism industry is of great significance for the transformation and upgrading of tourism. As a new tourism model integrated across industrial boundaries, the cultural and creative tourism complex is market-oriented, with “creativity” as the core, and deeply excavates the cultural connotation of tourism resources, reflecting a high degree of integration, creativity, and culture. It has broad market development prospects.

1. To encourage the growth of the creative economy, the government has released policies and improved the willingness of necessary finances

This essay contends that the primary factor influencing the growth of an innovative economy in developing nations is the government's policy backing. In order to develop cultural resources and tourism against the backdrop of the creative economy, the region should be based on the height of history, take into account the reality of the province's development, assess the situation, develop corresponding policies, and provide adequate financial support.

(2) Recognize the uniqueness of cultural resources and build tailored, high-quality tourism

When creating cultural resources, we must take into account the pertinent criteria of innovative economics, explore their uniqueness, and accurately account for their worth. In order to actualize the tourist development of cultural resources in the context of the creative economy, it is crucial to simultaneously construct high-quality scenic sites in order to prevent the growth of homogenization and convergence.

(3) The importance of developing the uniqueness of tourism resources and emphasizing the cultural diversity of the region

“Creativity” is the center of the innovation economy, and “innovation” itself is found in the pursuit of it. Therefore, the area should consider its richness and uniqueness when developing the tourism of cultural treasures. The findings demonstrate that the tourism development model based on cultural resources is a very effective strategy in the regional creative economy setting and has helped to advance regional economic growth. This is another example of how local cultural resources have grown in the context of the creative economy.

## Figures and Tables

**Figure 1:** The impact of tourism promotion.

**Figure 2:** The industrialization process of culture.

**Figure 3:** Representation of the vector space model.

**Figure 4:** Example diagram of recommendation principle of user-based collaborative filtering algorithm.

**Figure 5:** Evaluation results.

**Figure 6:** Influence results of various elements.

**Figure 7:** Comment feature results.

**Figure 8:** Comparison of scores of cultural tourism development results.

**Figure 9:** Tourist satisfaction evaluation.

**Table 1:** Yichun Scenic Area.

Area	Tourist attractions
Yuanzhou District	Yangshan Qiyin Temple
	Huacheng Temple
	Cihua Temple
	Yichun Chandu Cultural Expo Park
Shanggao County	Moshan Jiufeng Temple
Yifeng County	Huangbo Temple
	Dongsan Puri Temple
	Oriental Zen Cultural Park
Fengxin County	Baizhang Temple
Jing'an County	Baofeng Temple

**Table 2:** Division of Zen tourist attractions in Yichun.

Scenic spot	Product type and features
Yichun Chandu Cultural Expo Park, Yifeng County Oriental Zen Cultural Park	Cultural tourism, cultural experience; static display
Baizhang Temple, Baofeng Temple, Puli Temple, Qiyin Temple	Religious pilgrimage, cultural tourism, cultural experience, natural scenery sightseeing
Huangbo Temple, Jiufeng Temple	Religious pilgrimage
Huacheng Temple, Cihua Temple	Cultural tourism

**Table 3:** Words with more frequent occurrences in feature results.

Key feature serial number	Tourist batch 1	Tourist batch 2
2	Yichun Temple	Cultural park
7	Cultural teaching	Historical meaning
8	Free travel	Sun protection
9	Panoramic	Retro bokeh

## Data Availability

The data used to support the findings of this study are available from the corresponding author upon request.
